# An Analysis of the Cultivation Methods of Visual Communication Design in New Media Environment

This article has been retracted.

**DOI:** 10.1155/2022/2798019

**Published:** 2022-08-24

**Authors:** Meng Qi

**Affiliations:** Sookmyung Women's University, Department of Visual & Media Design, Seoul 04310, Republic of Korea

## Abstract

In order to better adapt to the teaching development needs of visual communication design in the new media environment, a method of visual communication design training based on the ecological environment of the new media environment is proposed. This method constructs a web-based professional course network teaching platform by cultivating practical design talents under the new platform, new environment, and new technology, starting from the perspective of practical application, starting from the teaching process of visual communication design specialty, combined with the needs of social development for students' creative needs, so as to provide rich visual communication design cases, design practice, and exchange and discussion platform for professional teaching. The results show that the local display time of the system page is too long. It takes 3.3 seconds to enter the query page manually, and the script test time is 0.3 seconds, so the page display time takes about 3 seconds. The system basically meets the functional requirements, but from the perspective of resource occupation, the program requirements are further optimized to reduce the utilization of CRU. From the analysis of memory usage, it is suggested to optimize the memory recycling mechanism.

## 1. Introduction

Visual communication is a special specialty. Its teaching focus is on self-confidence and cultivating innovative talents needed for all kinds of design for social development. Of course, communication design is not only focused on the area of new media, but also on the carrier of design [1]. However, compared with traditional media models, the new media environment places greater demands on students, requiring new ideas and innovations from students' education. Therefore, in the age of rapid development of information technology, the demand for intelligent technology in information communication as new media platforms is increasing. For schools and faculty, the training of communication designers is required to follow certain platforms, and at the same time, it is necessary to strengthen student intelligence [2]. However, from the current curriculum in this field, the professional setting is divided into the field of art, and basically all students majoring in art are carrying out professional education. Therefore, ecological environment of the professional design training of visual communication under the new media environment must pay attention to the cultivation of artistic esthetic ability and professional teaching.

## 2. Literature Review

The research on the current digital information education mode started earlier in this aspect, and now the development in this aspect has been at a high level, and the relevant development level and development mode of visual communication education have been continuously adjusted, so that it can adapt to the development of education in a long time [3]. When studying this aspect, it mainly focuses on some American companies. In the 1990s, new ways of visual communication education became popular in some countries such as Europe and the United States [4]. Some educators have proposed that this kind of visual education has changed the traditional educational concept, integrated the complete vision into the new educational model, changed the traditional teaching methods used in education with new knowledge and very important teaching objectives in education, took the knowledge and needs most concerned by students as the primary development condition in teaching, and formed a new way of education in the process of education [5]. This new way of education is to use visual communication to drive the development of education.

Some scholars pointed out that we should correctly grasp the goal and direction of multimedia development and take the corresponding theory and research basis as a level of development goal [6]. To realize the all-round development of digital multimedia, we should pay attention to the theoretical basis of this aspect, form the correct development direction, make an all-round prediction of the way of visual communication, and put forward that the unique characteristics and characteristics of art should be added to the visual communication design education, so as to add new vitality to the new development trend of education [7]. In terms of development direction, it is pointed out that the future development direction should be a diversified and diversified development direction, with the characteristics of good forms of visual communication design education [8]. It can be combined with some software. Through a large number of literature investigation and research, it is found that China's technical design level is still relatively backward in software design, which needs to be further improved, clarify the cultivation of artistic design and esthetic ability, master these two abilities, and combine visual elements in the overall education process of visual communication design.

The change in visual communication design naturally puts forward new requirements for design talents and design educators. The design can not only keep the graphic skills, or even complete the transmission of information, but also carry out communication design [9]. Therefore, designers first not only need to change their design ideas, master professional knowledge, and have esthetic ability, but also explore new expression methods and forms with new media as a bridge, and strive to become a new type of comprehensive talent. To achieve this goal, many colleges and universities are conducting research on educational reform, such as research on teaching practice, differentiation of teaching, the use of technology and integration, and the role of culture. Experience in teaching art design. For example, some colleges use the World University City network platform to develop resource plans to monitor resource allocation, support curriculum, and provide job training for some. This is a powerful exploration of the cultivation of industrial design talents in Higher Vocational Colleges under the background of informatization [10]. The other is that a university constructs a vocational post-oriented talent training mode based on information technology. These two studies are aimed at higher vocational education, and the construction of an information platform lacks the exertion of the characteristics of art and design specialty, and the strength of resource integration is not enough.

## 3. Visual Communication System Design

### 3.1. System Functional Requirements

According to the demand analysis of the system, the function of the whole website system is divided according to the idea of modular management [11]. The website system is divided into four subsystems: visual design case base, online course teaching, design project and work display, and design practice and communication, as well as supporting subsystems similar to user management and system management. The functional structure of the system is shown in Figure 1.

The use case diagram established by the visual case base is relatively simple, with only two roles: teachers and students. The main use cases include case upload, editing, deletion, browsing, retrieval, download, review, classified management, and release. Students can only upload cases, browse cases, retrieve cases, download cases, and edit their uploaded cases that have not passed the review. Teachers can also edit, delete, review, classify, manage, and publish cases.  Table 1 is the use case description of visual case retrieval.

Figure 2 is the use case diagram of online learning. This use case also has two roles: teachers and students. The main use cases include uploading teaching resources, course Q&A, online communication, course guidance, study guide, downloading materials, online learning, asking questions, and viewing question replies [11]. Students can download materials, online learning, online communication, course guidance, ask questions, view question replies, and teachers can upload teaching resources, course Q&A, online communication, study guide, and course guidance.  Table 2 is the use case description of teaching resources uploaded by teachers.

Figure 3 is the use case diagram of work evaluation. This use case also has two roles: teachers and students. The main use cases are work submission, online appreciation, online evaluation, evaluation item setting, and evaluation results. Teachers can carry out online appreciation, online evaluation, evaluation item setting, and evaluation results, and students can submit works, online appreciation, and online evaluation.  Table 3 is the use case description of evaluation item setting.

### 3.2. System Architecture Design

#### 3.2.1. Physical Architecture

The system takes the special campus network of the school as the network platform. The campus network has covered the teaching building, dormitory, and office building in the school. The backbone network system is Gigabit Ethernet [12]. The backbone network in each building adopts fast Ethernet technology and is interconnected with the school network center through optical cable to provide various network service functions. The physical architecture of the system is shown in Figure 4.

#### 3.2.2. Logical Architecture

The system adopts Microsoft's three-tier design idea, and the designed system architecture is shown in Figure 5. This architecture not only logically divides the functions of each module and the relationship between them, but also reflects the real component independence in physical implementation, which provides convenience for the separate maintenance and upgrading of client applications, web servers, and database servers in the future, and improves the flexibility of the system [13].

#### 3.2.3. Online Teaching Module Design

The online course teaching module includes learning guide, course guidance, teaching courseware, network course, and other functions. The teaching courseware module also includes courseware upload, courseware download, courseware retrieval, and other sub functions. Its functional structure is shown in Figure 6.

The online communication module includes online BBS, design practice, homework salon, and other columns. Its functional structure is shown in Figure 7.

BBS forum is set up in the system for communication between teachers and students, where students can discuss problems in teaching, put forward their own questions about the teaching content, the teacher can answer them online, and students can also discuss a topic [14]. Visual communication art design major attaches great importance to the cultivation of students' practical ability. Teachers establish a series of practical training projects on the website, including holiday greeting card production, game development, advertising production, website application, MV production, e-magazine, etc. For each training project, there are detailed descriptions of training objectives, basic knowledge, training equipment and environment, reference effect, reference effect production process, achievement evaluation method, submission content and method, etc. With reference to the production process, students can operate step by step and give full play to their creative ability. When evaluating students' projects, teachers not only focus on the results of the project, but also pay more attention to the creative process of students, and comprehensively analyze their comprehensive quality in the process of project design [15].

### 3.3. Detailed Design of the Course Teaching System

#### 3.3.1. System Content Modeling

The main task of the website system realized in this article is to provide online teaching resources, the functions of appreciation of various visual communication design works, submission and evaluation of students' works, as well as online communication and interaction, improve students' learning enthusiasm, supplement and extend the traditional teaching mode, and realize the purpose of resource and technology assisted classroom teaching on the platform of campus network. In this system, there are two important roles: teachers and students. Teachers are the people who mainly provide knowledge and resources, and students are the people who obtain knowledge and information and exchange ideas. The realization of their respective functions is discussed below.

#### 3.3.2. System Database Logic Design

E-R diagram is mainly a process of abstracting and summarizing the needs of users and abstracting entities and the relationships between entities. The relationship model is mainly in which the entities and the relationships between entities are represented by a single structure type, that is, relationship. When converting E-R diagram to relational diagram, we must fully consider whether the type of connection between entities is one-to-one, one to many, or many to many, and choose different conversion rules according to different types. After the system diagram is converted, the relationship table of the system can be obtained, which are introduced as follows [16].

Due to the large number of system data tables, each table contains too many attributes to be represented in a graph. We only extract the representative attributes of some entities and represent them with E-R graph. Through the demand analysis of the system database, we mainly analyze and establish “teacher information table,” “student information table,” “art work information table,” “website file information table,” “forum information table,” “question information,” “evaluation item information,” etc., the design methods of other information tables are the same.

Student table is used to save student information in the database. The table structure is shown in Table 4.

The problem table is used to save the problem information in the database. The table structure is shown in Table 5.

The art works table is used to store the art works information in the database. The table structure is shown in Table 6.

The website file table is used to store the website file information in the database. The table structure is shown in Table 7.

## 4. Optimization of Training Mode of Visual Communication Design Talents under the New Media Environment

### 4.1. Principles and Objectives of Mode Optimization

The new training mode emphasizes the development, sharing, and utilization of information in the process of talent training, and highlights the characteristics of informatization. The ultimate goal of this professional training is to promote the transmission of information through design works. Therefore, in the whole process of talent training, the concept of “through information, for information” is embodied, which is the concept that only the visual communication design specialty is most qualified to emphasize [17]. It can be expressed as information to information, or I2I mode for short (the conceptual diagram is shown in Figure 8).

The specific construction objectives are as follows:

- First, adjust the training objectives of professionals in combination with the impact of informatization on visual communication design. Analyze the demand of the times for talents, emphasize the importance of information literacy, and build a multi angle basic goal system of talent training, so as to better reflect the development needs of the times.
- Second, according to different teaching contents, we should comprehensively use traditional teaching, network teaching, and flipped classroom to improve students' autonomous learning ability, enrich the ways of interaction between teachers and students, open up students' learning channels, and improve teaching effect. By changing the teaching methods, on the one hand, follow up the social information exchange methods, and on the other hand, cultivate students' awareness and ability of lifelong learning.
- Third, build a professional information platform to realize the functions of social demand feedback analysis, teaching resource sharing, professional practice supply and demand communication, multi angle talent training evaluation, and so on [18].

### 4.2. Building Professional Information Platform to Ensure the Operation of Training Mode

#### 4.2.1. Construction of Information Platform

Firstly, we need to know how to allocate resources. Through the platform, we can understand the important status of education and training of related colleges and universities, obtain relevant information and experience, identify results that occur in the training process to ensure safety and appropriateness, and adopt additional policies of education and training. Through the platform, students can access curriculum information on key topics, including credit-accredited classes, and complete online courses and assessments. Obtain the auxiliary software and multimedia materials involved in the process of visual communication design and teaching, so as to facilitate further learning or creation. The social-oriented professional online open courses of colleges and universities can also be concentrated here for easy retrieval and use [19].

Secondly, information communication should be realized. On the basis of online course learning, the information platform provides a variety of interactive forms to realize real-time communication between teachers and students, improve teaching quality, and promote the improvement of communication and cooperation ability. Realize interschool professional exchanges through network platform, including professional lectures, teacher training, and design project cooperation. Realize the bidding of network design projects, job recruitment, information release and interaction of design competition information, and personal design needs [20].

Moreover, in order to realize the two functions of “resource collection” and “information interaction,” the platform needs to have the structure shown in Figure 9.

The platform includes six modules: security maintenance module, network teaching module, learning and creation resource module, information module, online communication module, and background support system. Each module is divided into several columns. First, through user authority management, we can automatically distinguish different identities such as ordinary visitors, teachers and students who log in, managers who can obtain application data, and ensure the smooth use of website resources. The network teaching module provides teachers and students with a networked, intelligent, and automatic and remote teaching environment and conditions. It provides necessary conditions for the realization of the flipped classroom, solves the remote guidance of enterprises to students in practice, facilitates Cross School credit, and plays the role of professional display. The learning and creation resource module provides guidance and helps for students' extracurricular extensible self-study, including software learning directly related to professional creation, multimedia materials required for creation, and literature, history, and philosophy resources to improve personal cultural cultivation [21]. The outstanding feature of the information module is rich and fast, which can provide the latest professional information, including professional development frontier, enterprise employment information, individual or group design needs, competition information, and the application status of visual communication design in life. The online communication module realizes information exchange and interaction in the form of forums, message boards, and other forms, and exists as an independent module or a subsidiary function of other modules. The background support system is the technical support of the whole platform, which is responsible for the operation and management of the website and the mining and utilization of the generated data resources.

In terms of platform technology application, give full play to and make use of mature technologies such as computer, Internet, mobile network, Internet of things, cloud computing, GPS and GIS, support mainstream computer software and hardware platforms, be compatible with existing equipment, and support a variety of open technology standards, which is conducive to system interconnection, mutual access, and expansion of application system functions. Realize the openness, operability, safety, and reliability of the system.

### 4.3. Integrating Design Education Resources to Improve Professional Practice Effect

#### 4.3.1. Practice Teaching System to Improve Practical Ability

“Practice course” is different from the design practice operation widely involved in professional skill courses. Practice module often refers to the independent practice class hours in the semester, mostly the practice experience separated from the school or classroom. Generally, the practice class hours of grade 1 and grade 2 are 4–6 weeks, and the practice class hours of grade 3 and grade 4 are 8–16 weeks. If conditions permit, the visual communication major should appropriately increase the practice class hours, especially for senior students, and provide sufficient time to exercise their practical ability [22].

The purpose of practical teaching in grade 1 and grade 2 is to integrate the foundation. In the past, the practice at this stage was mostly in the form of art style collection. The professional practice forms of visual communication should be rich and colorful, including lectures, exhibitions, visits, enterprise internships, etc., in order to understand the general situation of the industry and social needs. The key to practical courses lies in paying attention to practical results. We should make full use of every practical activity uniformly organized by the school, and let students make full preparations before listening to lectures and watching exhibitions, so as to make the visit more targeted. After the end of practical activities, we should also make a summary, so as to make the practical experience more profound and clear. In short, practice cannot be a mere formality [23].

The purpose of practical teaching in grade 3 and grade 4 is to improve the ability to solve problems. We should integrate the knowledge by completing the actual design project. However, in-depth company practice has always been a practice form that many colleges and universities sigh. There are many reasons for the difficulty in teaching and practical communication of visual communication design specialty. This problem can be effectively solved through the information platform.

#### 4.3.2. Practical Teaching Content Promotes Collaborative Innovation

Each course in the Professional Skills module should focus on design training as a key link to instruction in visual design. For a long time, college and university design communication classes were usually offered by instructors based on previous experience or developed by the students themselves. Only a handful of faculty and students of the top colleges and universities are involved in the real development projects. This is due to the fact that most graduates do not have enough design experience and it is difficult to adapt quickly to the needs of the job. At the same time, it is difficult to realize many people need design in real life, that is, design education cannot help people in real life and improve the level of relationships, good. Lack of access to general training is a hindrance to the development of this project. If we create a professional platform that can share multiple data resources, we can easily present a real project design. Through the information platform, share the details of communication visual design for communities and levels of capacity building of students, document the needs of companies and individuals people, and understand the information created to compete over time. According to the actual design ability of students, combined with the content of professional courses, the school can give full play to personal interests and expertise, and cooperate with relevant units to complete corresponding real projects through the platform.

The design projects in the course are completed according to the actual standards. Even if it is impossible to adopt every student's homework, it can greatly improve the teaching effect of practical training. Effectively broaden students' vision, improve students' practical ability and adaptability, and promote society's understanding and understanding of these professional design talents. More importantly, it can meet the development trend of the regional economy and the demand of the industry for talents. Among them, the information of professional platforms can play a key role in optimizing innovation resources [24].

### 4.4. Giving Full Play to the Ability of Independent Learning and Innovate Classroom Teaching Forms

#### 4.4.1. Activating Teaching Process

In reality, at present, students majoring in visual communication design need to do a lot of work after class to complete the professional course homework, including the understanding of the subject, the collection of data, and the production of finished products. Many of them are completed through the network. After all, we have been used to the exchange and application of network information in real life, but our professional course teaching process still stays in the past. There are many new forms of foreign classroom teaching reform, but in the social environment with the increasing degree of informatization, looking at these reforms and experiments, we have to admit that “flipped classroom” is more suitable for the majority of visual communication design in Colleges and universities. Flipped classroom is a class in which teachers write videos and students watch the teacher explain movies at home or outside the classroom, then return to the classroom to interact with the teacher and students and complete their homework. Compared with a traditional classroom, flipped classroom has many differences. Teachers change from knowledge imparters and classroom managers to learning instructors and promoters; students change from passive recipients to active researchers; the teaching process has changed from “classroom explanation + homework” to “pre-class learning + classroom guidance”; the main content in the classroom has changed from knowledge explanation to problem research; and the technology involved in teaching has changed from the content display on the blackboard or projection to the use of Internet Autonomous Learning and collaborative discussion tools. This learning process allows students to control the learning rhythm according to their own situation, which is convenient for review and in-depth learning, and helps to cultivate the habit and ability of autonomous learning. As a result, teachers have more guidance time and can give detailed guidance to the works one by one, so as to obtain a more ideal teaching effect. The form of flipped classroom is very consistent with the constructivist interpretation of the learning process and the definition of the roles of teachers and students. At present, many companies have developed relevant software programs, which are easy to operate and conducive to the realization of flipped classroom.

It is worth noting that vortex classes have not been extensively explored in communication visual design training courses today, largely due to the limited use of vortex classes, lecture. Currently, the subjects that are being tested in the classroom are specialized disciplines, while liberal arts education has many meanings, including the thoughts and ideas of the teachers, students, and will achieve better educational outcomes. In the past, majority of communication was found only in drama, and students graduated in literature. But now it is different. Not only has art evolved, but with the development of time, the concept of communication visual design has become more diverse, and it is not limited to art for a long time. Therefore, flipped classroom is also applicable to visual communication design. We just need to screen the courses, which are more suitable and which are not suitable. Compared with science courses, the teaching of visual communication needs to combine a large number of pictures, cases, audio, and video materials. Although the advantages of network information transmission can highlight the professional characteristics, it also puts forward higher requirements for teachers and servers. Teachers need to be able to synthesize various materials and make higher quality teaching videos, and need to provide high-performance servers to realize the application of flipped classroom in teaching.

#### 4.4.2. Mobilizing Sensory Experience

For example, in the professional basic courses to cultivate students' perception and creativity, most colleges and universities are used to following the modeling training methods of traditional art schools. In short, it is to describe and pursue painting which is not conducive to the exertion of creativity. As a result, our students cannot produce innovative works in the later stage. Therefore, the design market is rarely original and full of senseless plagiarism.

Mobilize students' own senses, make them full of keen perception of things, and try to express them in their own way, this will become a personalized expression. This is conducive to their understanding of the movement of light and trees in the classroom. It can also be used in the later stage of the classroom. Only in this way students can realize the great creativity contained in themselves and deliver colorful and sincere design. In addition, a lot of discussion in the visual communication design class in western countries is also a good way to cultivate students' divergent thinking. All these delicate guidances, on the one hand, can give full play to students' personality and expressiveness, at the same time, can make students not rely too much on computers in the creative process, and retain and develop their autonomy as human beings, which is also an aspect that is easy to be ignored and difficult and valuable in design education in the information age.

## 5. Conclusion

The main goal of visual communication is to develop new skills to meet the needs of building relationships. Both news and new media are carriers of communication design. Compared with traditional media design, new media requires new ideas and practices from students. Therefore, when the modern new media platform information communication industry is highly developed, teachers need to have certain platform characteristics and pay attention to students' ability to perform well, while teaching students communication. The concept of visual communication has continued since the turn of the century. Therefore, in some colleges and universities, especially in schools with poor teaching staff, there is a lack of professional development and openness to this position. Therefore, the school district should have a long-term growth plan for specialization in colleges and universities. Therefore, it is necessary for the department of education to have a future improvement plan to determine the size of the college. Many colleges and universities can provide training plans in key areas of education, learn new design concepts under the new era and new technology conditions in the ecological environment, and apply them to social needs, so as to make reasonable use and expansion of design thinking.

In short, with the continuous development of network media technology, mobile popular applications are the latest forms of communication channels. The teaching of visual communication majors in colleges and universities should carry out comprehensive training according to visual expression, information communication, and art design theory, focusing on the esthetic identification and ideological resonance of the communication audience. We should make good use of the advantageous operating environment of the new media platform to carry out effective communication, explore and practice according to the current psychological acceptance of the audience and the consumption needs, make visual communication gradually become the mainstream specialty in China's economic and social development, and provide technical support with artistic value for China's emerging industry chain.

## Figures and Tables

**Figure 1:** System function structure diagram.

**Figure 2:** Online student use case diagram.

**Figure 3:** Use case diagram of work evaluation.

**Figure 4:** System physical architecture.

**Figure 5:** System logic architecture.

**Figure 6:** Online course teaching function structure.

**Figure 7:** Design practice and communication function architecture.

**Figure 8:** Conceptual diagram of I2I talent training mode.

**Figure 9:** Structure of the professional information platform.

**Table 1:** Use case description of visual case retrieval.

Case number	QRY01 priority middle edition 1.0
Case name	Retrieval of visual case base
Brief description	View visual cases that match a keyword
Basic/typical process	1. The user enters the retrieval page of the visual case base
	2. Enter search keywords
	3. Click query
Optional/abnormal process	The query results are displayed on the page
Results of enforcement	Click query to display the following contents
	Case name, uploader, upload time, and case content

**Table 2:** Use case description of teaching resources uploaded by teachers.

Case number	SCHUAN01 priority middle edition 1.0
Case name	Upload teaching resources
Brief description	Teachers upload teaching resources to a course directory
Basic/typical process	1. The teacher enters the page of uploading teaching resources
	2. Select the course name of the resource
	3. Select the type of data: Type: Word document, video, PPT courseware, audio file
	4. Click upload
Optional/abnormal process	Teaching resources uploaded successfully
Results of enforcement	Click upload to display the following contents:
	Name, type and upload time of uploaded data

**Table 3:** Use case description of evaluation item setting.

Case number	PJIASET priority middle edition 1.0
Case name	Set evaluation items for submitted works
Brief description	Teachers set the evaluation indicators and proportion of works submitted by students
Basic/typical process	1. The teacher enters the evaluation item setting page
	2. Select students' works
	3. Click the evaluation item setting button
	4. Click the evaluation item setting and select the evaluation item to be included
	5. Set the effective start and end time of evaluation and the proportion of evaluation between teachers and students
	6. Click finish
Optional/abnormal process	Set successfully
Results of enforcement	Generate evaluation form

**Table 4:** Student information.

Field name	Field type	Field length	Explain
Id	Auto number	4	Primary key
Userid	Char	15	
Usemame	Char	20	
Userpwd	Char	20	
Usersex	Int	2	
Usercontact	Char	60	
Usergrade	Char	20	
Usermaior	Char	20	

**Table 5:** Problem information.

Field name	Field type	Field length	Explain
Id	Auto number	4	Primary key
Title	Char	15	
Content	Char	100	
Author	Char	20	
Replynums	Int	4	
Key	Char	30	
Time	Date		

**Table 6:** Information of art works.

Field name	Field type	Field length	Explain
Id	Auto number	4	Primary key
Sernum	Int	4	
name	Char	20	
Author	Char	20	
Position	Char	30	
Sort	Char	30	
Time	Date		
Key	Char		
Nums	Int		
Commend	Bool		

**Table 7:** Website file information.

Field name	Field type	Field length	Explain
Id	Auto number	4	Primary key
name	Char	30	
Title	Char	20	
Author	Char	20	
Time	Date		
Sort	Char	30	
Status	Char	20	
K	Char	100	
NRBeadnums	Int	4	

## Data Availability

The labeled data set used to support the findings of this study is available from the author upon request.
